RETRACTED

# MicroRNA-20a-5p promotes colorectal cancer invasion and metastasis by downregulating Smad4

**DOI:** 10.18632/oncotarget.9900

**Published:** 2016-06-07

**Authors:** Dantong Cheng, Senlin Zhao, Huamei Tang, Dongyuan Zhang, Hongcheng Sun, Fudong Yu, Weiliang Jiang, Ben Yue, Jingtao Wang, Meng Zhang, Yang Yu, Xisheng Liu, Xiaofeng Sun, Zongguang Zhou, Xuebin Qin, Xin Zhang, Dongwang Yan, Yugang Wen, Zhihai Peng

**Affiliations:** ^1^ Department of General Surgery, Shanghai General Hospital, School of Medicine, Shanghai Jiao Tong University, Shanghai, China; ^2^ Department of Pathology, Shanghai General Hospital, School of Medicine, Shanghai Jiao Tong University, Shanghai, China; ^3^ Department of Pathology, Fudan University Affiliated Shanghai Cancer Center, Shanghai, China; ^4^ Department of Gastroenterology, Shanghai General Hospital, School of Medicine, Shanghai Jiaotong University, Shanghai, China; ^5^ Department of Oncology and Department of Clinical and Experimental Medicine, Linköping University, Linköping, Sweden; ^6^ Department of Gastrointestinal Surgery, West China Hospital, Sichuan University, Chengdu, Sichuan, China; ^7^ Department of Neuroscience, School of Medicine, Temple University, Philadelphia, PA, USA; ^8^ Department of Pathology, Zhejiang Provincial People's Hospital, Hangzhou, Zhejiang, China

**Keywords:** miR-20a-5p, colorectal cancer, metastasis, prognosis, Smad4

## Abstract

**Background:**

Tumor metastasis is one of the leading causes of poor prognosis for colorectal cancer (CRC) patients. Loss of Smad4 contributes to aggression process in many human cancers. However, the underlying precise mechanism of aberrant Smad4 expression in CRC development is still little known.

**Results:**

miR-20a-5p negatively regulated Smad4 by directly targeting its 3′UTR in human colorectal cancer cells. miR-20a-5p not only promoted CRC cells aggression capacity *in vitro* and liver metastasis *in vivo*, but also promoted the epithelial-to-mesenchymal transition process by downregulating Smad4 expression. In addition, tissue microarray analysis obtained from 544 CRC patients’ clinical characters showed that miR-20a-5p was upregulated in human CRC tissues, especially in the tissues with metastasis. High level of miR-20a-5p predicted poor prognosis in CRC patients.

**Methods:**

Five miRNA target prediction programs were applied to identify potential miRNA(s) that target(s) Smad4 in CRC. Luciferase reporter assay and transfection technique were used to validate the correlation between miR-20a-5p and Smad4 in CRC. Wound healing, transwell and tumorigenesis assays were used to explore the function of miR-20a-5p and Smad4 in CRC progression *in vitro* and *in vivo*. The association between miR-20a-5p expression and the prognosis of CRC patients was evaluated by Kaplan–Meier analysis and multivariate cox proportional hazard analyses based on tissue microarray data.

RETRACTED

**Conclusions:**

miR-20a-5p, as an onco-miRNA, promoted the invasion and metastasis ability by suppressing Smad4 expression in CRC cells, and high miR-20a-5p predicted poor prognosis for CRC patients, providing a novel and promising therapeutic target in human colorectal cancer.

## INTRODUCTION

Although clinical diagnosis and therapies have achieved much progress with the improvement of surgical and medical treatments, the prognosis of CRC patients is still not optimistic [1]. The poor follow-up is mainly caused by the tumor metastasis or recurrence [2]. Therefore, it is urgently essential to reveal the underlying molecular mechanism of CRC metastasis progression for refining therapeutic strategies.

Drosophila mothers against decapentaplegic protein4 (Smad4) is the central critical signal transduction element of the transforming growth factor (TGF–β) superfamily. Smad4 mutation brings about the functional switch of TGF–β from tumor suppressor to tumor promoter, driving aggression in many human cancers [3]. For example, in gastric adenocarcinomas developed lung metastases, loss of Smad4 accumulates nuclear β–catenin, resulting in β-catenin target genes MMP7 and Vimentin overexpressing thus promoting epithelial-to-mesenchymal transition [4]. In glioblastoma, inactivation of Smad4 can enhance self-renewal capacity of tumor-derived spheroids *in vitro*, depending on downregulating Id1 and Id3 expression [5]. In colon cancers, loss of Smad4 promotes colorectal cancer progression by accumulation of myeloid-derived suppressor cells through the CCL15-CCR1 chemokine axis in an orthotropic xenograft model [6]. Recently, increasing researches have revealed some miRNAs directly regulated the expression of Smad4 in tumor aggression. miR-224, as an oncogenic miRNA, facilitates tumor progression by shifting the equilibrium of the partially antagonist functions of SMAD4 toward enhanced invasion and growth in non-small-cell lung cancer [7]. Overexpression of miR-301a-3p inhibits the target gene Smad4, enhancing pancreatic ductal adenocarcinoma (PDAC) cells colony, invasion and migration abilities *in vitro* as well as tumorigenesis *in vivo* [8]. Therefore, it is well worth to explore the interaction between Smad4 and miRNAs and the precise mechanism in CRC development.

miRNAs are small non-coding RNAs (18–25nt) which bind to the sequence-complementary of 3′untranslated region (3′UTR) of the target mRNAs, resulting in degradation or translational inhibition of target mRNAs. According to their targets, miRNAs are divided into onco-miRNAs and suppressors in cancers [9]. Certain aberrant miRNAs have been discovered involved in CRC. For example, lower miR-497 levels in human CRC tissues induce KSR1 expression which is associated with CRC cancer occurrence, advanced stages, metastasis and chemoresistance [10]. miR-409–3p is a metastatic suppressor, and endogenous expression analysis revealed post-transcriptional inhibition of the onco-protein GAB1 is one of the mechanisms of action of this miRNA in CRC cells [11]. miR-181a-5p inhibits colon cancer cell migration and angiogenesis via downregulation of matrix metalloproteinase-14 [12]. Although these miRNAs have been discovered the important role in CRC development, there is still a sensitivity limitation applying to clinical diagnosis and treatment. Therefore, it's essential to search for novel and efficient miRNAs markers for CRC patients.

RETRACTED

Given the importance of miRNAs and Smad4 in cancers’ development, herein we seek to discover novel miRNAs which are able to regulate Smad4 in CRC. Here, we identified a novel miRNA, miR-20a-5p, which targeted smad4 3′-UTR, and verified that 1) high miR-20a-5p expression promoted the invasion and metastasis of CRC cells and induced EMT of CRC cells by directly binding to the 3′-UTR of Smad4; 2) most importantly, we also revealed that miR-20a-5p was upregulated in CRC tissues and high miR-20a-5p expression predicted the poor prognosis. Taken together, miR-20a-5p/Smad4 signal pathway may be a promising therapeutic target for CRC patients.

## RESULTS

### miR-20a-5p negatively regulated Smad4 in human colorectal cancer

miRanda, TargetScan, PicTar, RNA22 and PITA, these five miRNA target prediction programs were applied to identify potential miRNA(s) that target(s) Smad4 3′UTR. Only miRNAs binding to the same region in the target 3′-UTR sequence in at least three programs, were selected in following experiments. As shown in Supplementary Table 1, it was observed that 17 miRNAs had the same potential binding site to the 3′-UTR of Smad4. To identify the effect of these miRNAs on the expression of Smad4, miRNA mimics and luciferase reporter construct containing wild-type Smad4 3′-UTR were co-transfected into 293T cells. Transfection with miR-34c-5p, -17-5p, -19a-3p, -20a-5p, -19b-3p, -454-3p, -301a-3p, -106b-5p, -20b-5p, -106a-5p and -130a-3p mimics showed downregulated luciferase activity compared with transfection with normal control (NC)(Figure 1A). Among these, miR-20a-5p whose robust downregulation effect drew our attention, indicating that miR-20a-5p may be the most powerful potential regulator of Smad4 in these 17 miRNAs.

RETRACTED

**Figure 1:** miR-20a-5p negatively regulated Smad4 in human colorectal cancer (**A**) 293T cells were co-transfected with the negative control (NC) or miRNA mimics and the luciferase reporter construct containing the wild-type Smad4 3′-UTR. The luciferase activity of the NC was set to 1, the others were normalized to the NC. *P < 0.05 was considered to be statistically significant. (**B** and **C**) The mRNA expression of miR-20a-5p (*P* = 0.0002) and Smad4 (*P* < 0.001) in 10 CRC patients’ tissues with and without metastasis was evaluated by qRT-PCR. (**D**) The correlation between miR-20a-5p and Smad4 mRNA expressions in 10 colorectal cancer patients was evaluated using Spearman's correlation analysis (*P* = 0.031, R^2^ = 0.234). (**E**) The expression of miR-20a-5p in different colorectal cancer cells was evaluated by qRT-PCR. FHC was used as a control. (**F**) HT29 cells were infected with miR-20a-5p-expressing lentiviral vector and HCT116 cells were infected with miR-20a-5p-knockingdown lentiviral vector. The luciferase reporter construct containing the wild-type Smad4 3′-UTR. Empty vector was used as a control, *P < 0.05. (**G**) The expression levels of Smad4 mRNA and protein were evaluated using qRT–PCR and western blot analysis in empty vector-infected or miR-20a-5p vector infected HT29 cells and negative control or anti-miR-20a-5p vector infected HCT116 cells, respectively, *P < 0.05.

Subsequently, we evaluated miR-20a-5p and relative Smad4 expression level in 10 patients’ colorectal cancer tissues with and without metastasis. We found that miR-20a-5p was significantly upregulated (Figure 1B, *P* = 0.002), while Smad4 was obviously downregulated (Figure 1C, *P* < 0.001) in tissues with metastasis than those without metastasis. What's more, the expression of miR-20a-5p was negatively correlated with that of Smad4 in these 10 patients (Figure 1D, R^2^ = 0.234, *P* < 0.001). To further validate the role of miR-20a-5p and Smad4 in CRC, eight colorectal cell lines and one normal colorectal epithelial cell line were used for testing the relative expression of miR-20a-5p. Compared with the normal colon epithelial cell line (FHC cell line), HCT116 cell line which owned high ability of migration and invasion as previously proved [13], showed high expression level of miR-20a-5p, while the low migration and invasion ability cell line HT29 performed low expression level of miR-20a-5p (Figure 1E). Then HCT116 and HT29 cell lines were selected for further studies. After transfecting miR-20a-5p mimics and anti-miR-20a-5p mimics into HT29 and HCT116 cell line respectively, we found miR-20a-5p mimics inhibited Smad4 3′-UTR luciferase activity in HT29 cells, conversely, anti-miR-20a-5p mimics promoted Smad4 3′-UTR luciferase activity in HCT116 cells (Figure 1F, *P* < 0.05), which demonstrated that miR-20a-5p might directly target the 3′-UTR of Smad4 in CRC cell lines. Furthermore, we found miR-20a-5p repressed Smad4 expression at mRNA and protein level (Figure 1G, *P* < 0.05). All the above results suggested that miR-20a-5p was a negative regulator of Smad4 in human colorectal cancer.

RETRACTED

### miR-20a-5p promoted invasion and metastasis of colorectal cancer cells *in vitro* and *in vivo*

To explore the function of miR-20a-5p in CRC progression, firstly, we performed wound healing assay and transwell assay *in vitro*. Overexpressing miR-20a-5p promoted the migration and invasion ability in HT29 cells (Figure 2A–2C, *P* < 0.01 for all), while knocking-down miR-20a-5p suppressed the migration and invasion ability in HCT116 cells (Figure 2A–2C, *P* < 0.01for all). These results indicated miRNA-20a-5p could promote CRC aggression *in vitro*. Then, we conducted the vivo assay in nude mice. HT29 cells with stable miR-20a-5p overexpression and HCT116 cells with stable miR-20a-5p silenced expression were injected into the nude mice from the tail's veins, and the control groups were injected with the same number and concentration of cells transfected with empty lentiviral vectors. We compared the colonies formed in the livers of the mice and found that miR-20a-5p overexpression or knocking-down could significantly increase or decrease the liver metastatic colonies compared with the control (Figure 2D, *P* < 0.001). These data further demonstrated that miR-20a-5p overexpressing cells were more powerful of liver metastatic colonies. Overall, these findings suggested miR-20a-5p could increase the invasion and metastasis ability of colorectal cancer cells *in vitro* and *vivo*.

**Figure 2:** Up-regulated miR-20a-5p promoted the invasion and metastasis of colorectal cancer *in vitro* and *in vivo* (**A**) Wound healing assay (**B**) Migration and (**C**) invasion assays were performed both in empty vector-infected or miR-20a-5p vector infected HT29 cells and negative control or anti-miR-20a-5p vector infected HCT116 cells, respectively. The results were presented as the mean ± SD of values.(A) The “wound” was created in a cell monolayer, and captured the images at the beginning and at 48 h. Compared the images to quantify the closed rate of the cells,**P < 0.01.(B and C) The number of cells that passed through the membrane was counted in 10 fields (**P < 0.01, magnification ×200). (**D**) Impact of miR-20a-5p on tumor metastasis *in vivo*. The number of metastatic liver colonies was counted. The images of normal liver tissue (1) and metastatic colony tissue (2) stained by HE were presented (***P < 0.001, magnification × 200).

RETRACTED

### miR-20a-5p promoted epithelial-to-mesenchyme transition of colorectal cancer cells

Increasing studies have proved that epithelial–mesenchyme transition (EMT) acted as the important step in metastatic dissemination of cancer cells, characterized by loss of cell-cell adhesion and gain of migratory and invasive capabilities [14]. Interestingly, there were obvious phenotypic changes in miR-20a-5p overexpressing HT29 cells and miR-20a-5p knocking-down HCT116 cells, compared with the control groups. Overexpressing miR-20a-5p induced mesenchyme phenotype alteration in HT29 cells, while knocking-down miR-20a-5p tended to epithelial cell phenotype in HCT116 cells (Figure 3A). Further, qRT-PCR assay showed the mesenchyme cell marker N-cadherin mRNA was significantly upregulated (*P* < 0.01) and the epithelial marker E-cadherin mRNA was significantly downregulated (*P* < 0.01) in HT29 cells upon miR-20a-5p overexpression (Figure 3B), whereas the mRNA of E-cadherin was upregulated (*P* < 0.01) and N-cadherin was downregulated (*P* < 0.05) in HCT116 cells upon miR-20a-5p knocking-down (Figure 3B). The similar changes of E-cadherin and N-cadherin were also found at protein level (Figure 3C). Taken together, miR-20a-5p could promote EMT process of CRC cells.

**Figure 3:** miR-20a-5p promoted the epithelial-to-mesenchymal transition of colorectal cancer cells (**A**) The alteration of phenotypic observed under microscopy (magnification × 200) in miR-20a-5p overexpressing HT29 cells and miR-20a-5p knocking-down HCT116 cells. (**B**) Expression of E-cadherin and N-cadherin were evaluated at mRNA and protein levels (*P < 0.05, **P < 0.01).

### miR-20a-5p mediated Smad4 expression by directly binding to its 3′-UTR

For negative regulation on Smad4, we further investigated whether Smad4 was the direct target of miR-20a-5p. We found wild type Smad4 3′-UTR mRNA contained a length of sequence conserved miR-20a-5p and conducted mutant miR-20a-5p and conserved mutant Smad4 3′-UTR, so miR-20a-5p with the complementary Smad4 3′UTR sites were mutated as reported previously [35, 36] (Figure 4A). Double-luciferase reporter system was used to validate our expectation. Figure 4B showed miR-20a-5p overexpression remarkably suppressed the luciferase activity of the wild-type Smad4 3′-UTR luciferase construct (Figure 4B *P* < 0.05) but not the mutant Smad4 3′UTR. Meanwhile, mutant-miR-20a-5p expression had no influence on the luciferase activity of wild-type Smad4 3′-UTR but can alter the mutant Smad4 3′-UTR luciferase activity (Figure 4B *P* < 0.05) in HT29 cells. On the contrary, both knockdown of miR-20a-5p and mutant-miR-20a-5p expression can promote luciferase activity of the wild-type Smad4 3′-UTR luciferase construct (*P* < 0.01) as well as mutant-type Smad4 (Figure 4C *P* < 0.001). Taken together, miR-20a-5p mediated Smad4 expression by directly targeting its 3′-UTR, which may be involved in the promoting role in CRC progression.

RETRACTED

**Figure 4:** miR-20a-5p mediated Smad4 expression by directly binding to its 3′-UTR in CRC cell lines (**A**) The complementary sequences between the position 1357–1363 of wild-type or mutant human Smad4 3-UTRs mRNA and human miR-20a-5p. (**B**) HT29 cells were co-transfected with the control vector, miR-20a-5p or mutant miR-20a-5p mimics and the luciferase reporter construct containing the wild-type or mutant Smad4 3′-UTR. (**C**) HCT-116 cells were co-transfected with the negative control, anti-miR-20a-5p or mutant-miR-20a-5p mimics and the luciferase reporter construct containing the wild-type or mutant Smad4 3′-UTR. For each experiment, the results were normalized to the luciferase activity detected in the cells transfected with the control vector. (*P < 0.05 **P < 0.01 ***P < 0.001).

### miR-20a-5p promoted the onco-process of CRC cells via Smad4 repression

Having shown the metastasis-promoting function of miR-20a-5p and its direct targeting role on Smad4, we further validated the biological function of Smad4 in the CRC aggression process mediated by miR-20a-5p. Consistent with the previous studies, overexpression or loss of Smad4 inhibited or promoted metastasis in CRC cells (Figure 5A, 5B *P* < 0.05). Further, in HT29 cells, as shown, overexpressing miR-20a-5p promoted wound healing and migration-invasion capacity *in vitro* and more liver metastatic colonies *in vivo*, but the effect was partially weakened after increasing Smad4 expression (Figure 5A *P* < 0.05). In HCT116 cells, the suppression effect of invasion and metastasis capacity *in vitro* and *in vivo* by knocking-down miR-20a-5p could be partially restored after silencing Smad4 expression (Figure 5B *P* < 0.05). What's more, overexpression or knocking-down of Smad4 could also partially reverse the roles of miR-20a-5p in EMT process (Figure 5C *P* < 0.05, Figure 5D). All these results indicated that Smad4 was a direct functional target of miR-20a-5p in aggression process in CRC cells.

**Figure 5:** miR-20a-5p promoted the onco-process of CRC cells via Smad4 repression miR-20a-5p overexpressing and negative control HT29 cells were transfected with empty vectors or Lv-Smad4. miR-20a-5p knocking down and negative control HCT-116 cells were transfected with empty vectors or shSmad4. (**A**) Wound healing assay, migration and invasion assays were performed in HT29 cells. Smad4 overexpression partially abrogated the increased wound healing, invasion and metastasis capacity induced by upregulation of miR-20a-5p. (**B**) Wound healing assay, migration and invasion assays were performed in HCT116 cells. Smad4 knockdown partially restored the decreased wound healing, invasion and metastasis capacity induced by downregulation of miR-20a-5p. (**C**) The expression level of E-cadherin and N-cadherin mRNA was evaluated by qRT-PCR. Overexpression or knockdown of Smad4 partially reversed the promoted or inhibited EMT due to miR-20a-5p upregulation or downregulation. (**D**) The expression level of E-cadherin and N-cadherin protein was evaluated by western blot analysis. (**E**) The number of tumor colonies formed in animal models. Overexpression or knockdown of Smad4 partially reversed the number of liver metastatic colonies resulting from miR-20a-5p upregulation or downregulation. (*P < 0.05; **P < 0.01, ***P < 0.001).

RETRACTED

### High level of miR-20a-5p was correlated with the metastasis and predicted poor prognosis in colorectal cancer patients

To further investigate the clinical role of miR-20a-5p and Smad4, tissue microarray including 544 CRC patients was used to the following study. The clinical characters of these patients and their correlated miR-20a-5p and Smad4 protein expression levels were shown in Table 1. Compared with adjacent normal tissues, miR-20a-5p was upregulated and Smad4 was downregulated obviously in colorectal cancer tissues (Figure 6A, 6C1–6C3, *P* < 0.001). What's more, tumor metastasis patients showed a higher miR-20a-5p while lower Smad4 expression level than those without tumor metastasis (Figure 6B, 6C2–6C3, *P* < 0.001). Statistical analyses showed 74.8% (407/544) patients performed high expression of miR-20a-5p and 70.0% (381/544) patients showed low expression of Smad4 (Table 1A). High miR-20a-5p expression was positively correlated with pT stage (*P* = 0.035), pN stage (*P* = 0.001), pM stage (*P* = 0.022), American Joint Committee on Cancer (AJCC) stage (*P* = 0.005), differentiation (*P* = 0.022), and Smad4 (*P* < 0.001). While there were no significant relationships with patients’ age (*P* = 0.076), gender (*P* = 0.693) and tumor location (*P* = 0.280) (Table 1A). What's more, low Smad4 expression level was also negatively correlated with pT stage (*P* = 0.004), pN stage (*P* = 0.006), pM stage (*P* = 0.032), and AJCC stage (*P* = 0.044), not with patients’ age (*P* = 0.773), gender (*P* = 0.779), tumor location (*P* = 0.124), and differentiation (*P* = 0.255) (Table 1A). These indicated that high miR-20a-5p and low Smad4 played significant roles in the patients’ tumor progress and may be valuable in prognostic prediction.

RETRACTED

**Table 1:** Relationship between clinical features and miR-20a-5p or Smad4 protein expression in 544 colon cancer patients

	miR-20a-5p expression		p*	Smad4 expression		p*
	Low (*n* = 137)	High (*n* = 407)		Low (*n* = 381)	High(*n* = 163)	
Age						
< 65	54 (39.4)	154 (37.8)	0.761	144 (37.8)	64 (39.3)	0.773
≥ 65	83 (60.6)	253 (62.2)		237 (62.2)	99 (60.7)	
Gender						
Female	37 (53.3)	207 (50.9)	0.693	198 (52.0)	82 (50.3)	0.779
Male	64 (46.7)	200 (49.1)		183 (48.0)	81 (49.7)	
Location						
Right	37 (27.0)	87 (21.4)	0.280	82 (21.5)	42 (25.8)	0.124
Transverse	9 (6.6)	24 (5.9)		19 (5.0)	14 (8.6)	
Left	91 (66.4)	296 (72.7)		280 (73.5)	107 (65.7)	
pT stage						
T1–2	38 (27.7)	79 (19.4)	0.035*	68 (17.9)	49 (30.1)	0.004*
T3–4	99 (72.3)	328 (80.6)		313 (72.1)	114 (70.0)	
pN stage						
N0	93 (67.9)	221 (54.3)	0.001*	209 (54.9)	105 (64.4)	0.006*
N1–2	44 (32.1)	186 (45.7)		172 (45.1)	58 (35.6)	
pM stage						
M0	133 (97.1)	371 (91.2)	0.022*	347 (91.1)	157 (96.3)	0.032
M1	4 (2.9)	36 (8.8)		34 (8.9)	6 (3.7)	
AJCC stage						
I–II	91 (66.4)	210 (51.6)	0.005*	198 (52.0)	103 (63.2)	0.044*
III–IV	46 (33.6)	197 (49.4)		183 (48.0)	60 (36.8)	
Differentiation						
Well	37 (27.0)	79 (19.4)	0.022*	76 (19.9)	40 (24.5)	0.255
Moderate	86 (62.8)	250 (61.4)		235 (61.7)	101 (62.0)	
Poor	14 (10.2)	78 (19.2)		70 (18.4)	22 (13.5)	
Smad4						
Negative	24 (17.5)	357 (87.7)	< 0.001*			
Positive	113 (82.5)	50 (12.3)				

* *p* < 0.05 indicates a significant relationship among the variables;

AJCC, American Joint Committee on Cancer.

**Figure 6:** High level of miR-20a-5p was correlated with the metastasis and predicted poor prognosis in colorectal cancer patients (**A**) The expression of miR-20a-5p mRNA in 544 patients normal and paired tumor tissues through qRT-PCR (*P* < 0.001). (**B**) The expression of miR-20a-5p mRNA in metastasis and non-metastasis tumor tissues. (**C**) The expression of Smad4 protein in tissues through IHC staining method: C1 normal tissue with low miR-20a-5p and Smad4 strong staining; C2 non-metastasis tumor tissue with high miR-20a-5p and Smad4 moderated staining, C3 metastatic tumor tissue with high miR-20a-5p and Smad4 weak staining. (**D**) Disease free survival (DFS) and (**E**) overall survival (OS) rates in 544 patients by Kaplan–Meier analysis with log-rank test (**P < 0.001). (F and G) overall survival (OS) rates in patients with tumor relapse (*P* = 0.003) and without tumor relapse patients (*P* = 0.547) by Kaplan–Meier analysis with log-rank test.

Subsequently, Kaplan–Meier analysis with log-rank test showed high miR-20a-5p expression patients presented poorer disease free survival (DFS) and overall survival (OS) rates than those with low miR-20a-5p expression (Figure 6D, 6E, *P* < 0.001). Further OS survival analysis showed that high level of miR-20a-5p in patients with tumor relapse also performed shorter survival time (Figure 6F, *P* = 0.003), while, there was no significant difference seen in the patients without tumor relapse (Figure 6G, *P* = 0.574). What's more, Multivariate cox proportional hazard analyses also revealed that advanced TNM stage and high miR-20a-5p expression contributed to poor DFS and OS (Table 2 *P* < 0.05 for all). Totally, high level of miR-20a-5p predicted poor prognosis of CRC patients, especially for patients with tumor recurrence.

RETRACTED

**Table 2:** Multivariate Cox proportional hazard analyses of miR-20a-5p expression and TNM in 544 CRC patients’ DFS and OS

Factors	Multivariate Analyses (DFS)		Multivariate Analyses (OS)	
	HR (95% CI)	P*	HR (95% CI)	P*
T stage (T3–4 vs T1–2)	1.60 (1.32–1.93)	< 0.001	1.54 (1.28–1.86)	< 0.001
N stage (N1–2 vs N0)	1.41 (1.17–1.70)	< 0.001	1.34 (1.11–1.61)	0.002
M stage (M1vs M0)	2.71 (1.80–4.06)	< 0.001	2.71 (1.80–4.06)	< 0.001
miR-20a-5p expression	7.90 (4.30–14.53)	< 0.001	8.22 (4.47–15.12)	< 0.001

* *P* < 0.05 indicates significance; HR, hazard ratio; CI, confidence interval.

## DISCUSSION

Previous studies have revealed that loss of Smad4 is seen in 30%–40% CRC patients [15], occurs late in the adenoma-to-carcinoma sequence [16], and contributes to liver metastases, a poor response to chemotherapy followed with poor prognosis [17, 18]. In our study, we identified a novel miRNA, miR-20a-5p, which could directly target Smad4 3′UTR in CRC cells and cause its downregulation. Further we demonstrated that miR-20a-5p promoted CRC cells invasion and metastasis by repressing Smad4 *in vitro* and *vivo*. In addition, high miR-20a-5p predicted poor prognosis for CRC patients. Thus miR-20a-5p may be an efficient marker for predicting the prognosis of the CRC patients and patients with high miR-20a-5p level might receive the stronger and individual treatment after surgery.

The occurrence of invasion and metastasis after operation is the leading cause of poor prognosis for CRC patients [19]. Dysregulated miRNAs were involved in CRC aggression. MicroRNA-17–5p promotes tumor metastasis of colorectal cancer by repressing PTEN expression [20]. Quantitatively controlling expression of miR-17–92 determines colon tumor progression in a mouse tumor model [21]. Because of the important tumor-suppressor role of Smad4 in CRC, we attempted to identify novel miRNAs which regulated Smad4 in tumorgenesis and metastasis process. miR-20a-5p has been reported to play a significant role in gastric cancer, non-small cell cancer, prostate cancer and other cancers. High level of miR-20a-5p generally indicates advanced stage, poor prognosis and chemo-therapy resistance in several cancer types. As for CRC, previous study revealed that combined the other five miRNAs (miR-21–5p, miR-103a-3p, miR-106b-5p, miR-143–5p, and miR-215), their prognostic and predictive role in predicting which patients benefit from adjuvant chemotherapy for stage II colon cancer [25], while the role of miR-20a-5p have not been explored in CRC yet. Hence, we tried to explore the function of miR-20a-5p in colorectal cancer development and we confirmed that miR-20a-5p was upregulated in CRC tissues, especially metastatic tissues than non-metastatic tissues. Not only in CRC, in breast cancers, miR-20a-5p with miR-17–5p and miR-18a-5p, were also increased in triple-negative compared with the luminal A [22]. In nasopharyngeal carcinoma, overexpressed miR-20a-5p combined with miR-24–3p, miR-891a, miR-106a-5p and miR-1908 formed the exosomes to downregulated the MARK1 signaling pathway to alter cell proliferation and differentiation [23]. Similarly, our studies also demonstrated overexpressing miR-20a-5p promoted CRC cells invasion and metastasis *in vitro* and more liver metastatic colonies *in vivo*.

RETRACTED

EMT has been validated an important step involved in invasion and metastasis process. During EMT process, cells lose these epithelial characteristics, gaining instead an invasive and migratory mesenchymal phenotype, which permits these cells to leave the tissue parenchyma and enter the systemic circulations during cancer metastasis [14, 24]. Herein, upregulated miR-20a-5p was also found inducing the mesenchyme phenotype alteration and increased mesenchyme cell marker N-cadherin and decreased epithelial marker E-cadherin expression, while downregulated miR-20a-5p manifested reverse performances in CRC cells. More importantly, with tissue microassay including 544 CRC patients analyses, we also validated that high level miR-20a-5p of CRC patients performed advanced stage and short survival time, suggesting miR-20a-5p could be an independent prognosis predictor for CRC patients. These discoveries further demonstrated the oncogenic role of miR-20a-5p in CRC.

Onco-miRNAs play the role in cancer progression by downregulating the expression of targeting tumor suppressors [26, 27]. Smad4, functions as common partner Smad4 (co-Smad4), once TGF-β binds to its receptor, and binds with phosphorylated Smad2/3 to form transcription complex and regulates the target gene expression [28, 29]. Smad4 mutation and downregulation contributes to many cancers progression. Smad4 deletion developed metastatic squamous cell carcinomas and correlated with EMT and lung metastasis in transgenic mice model [30]. Knockdown of SMAD4 partially conferred resistance to the anti-growth effects of BMP ligand in HCC cells and reduced the efficiency of colony formation and migratory capacity of HCC cells [31]. In the present, Smad4 was demonstrated to be a downstream target of miR-20a-5p in CRC progression. miR-20a-5p contained a length of specific converse binding sequence of Smad4. Further, functional studies demonstrated that overexpression of Smad4 partially abrogated the promoted invasion-migration-metastasis and EMT mediated by miR-20a-5p overexpression. Our findings suggested that miR-20a-5p promoted the onco-process of CRC cells by repressing Smad4 expression. In addition, patients with high miR-20a-5p expression usually showed a low Smad4 expression. Taken together, Smad4 played a significant role on the CRC progression mediated by miR-20a-5p. Based on the miRNA target prediction programs analysis, we only selected miR-20a-5p and identified Smad4 was the functional downstream target of miR-20a-5p in CRC progression, however, whether there existed other promising targets of miR-20a-5p in colorectal cancer progression needs more intensive researches.

RETRACTED

In summary, we identified a novel miRNA, miR-20a-5p, targeted Smad4 and promoted CRC invasion and metastasis. Interrupt or inhibiting the miR-20a-5p/Smad4 pathway may provide a novel therapeutic method for CRC patients. As miR-20a-5p had the predicting role on the chemosensitivity of stage II colorectal cancer [25], whether miR-20A-5p also predicted the chemosensitivity of other stage CRC patients is unknown and the specific mechanisms also need to be further explored.

## MATERIALS AND METHODS Figure and Tables

### Patients and tissue specimens

All the clinical specimens were obtained from 544 patients who have been diagnosed with colorectal cancer histologically from General Surgery Department, Shanghai General Hospital. All of the patients underwent surgical resection at between 2005 and 2011, and none of them have received neoadjuvant chemotherapy and radiation therapy before surgery. The 544 patients were divided into tumor recurrence and non-recurrence group. For surviving patients, the data were censored at the last follow-up. The patients’ clinic-pathologic characteristics characters were presented in Supplementary Table 2. Written informed consent was obtained from all patients, and the study was approved by the Ethics Committee of Shanghai General Hospital.

### Cell lines and nude mice

The cell line 293T cell, human colon mucosal epithelial cell line (FHC) and eight human colorectal cancer cell lines (HT29 SW480 LoVo DLD-1 HCT-8 RKO SW620 and HCT116) were purchased from Shanghai Institute of Biochemistry and Cell Biology, Chinese Academy of Sciences (Shanghai, China). Relative cell lines were generated from HT29 or HCT116 by transfection or lentivirus transduction following the manufacturer's instruction. These cells were cultured in a humidified 5% CO2 atmosphere at 37°C, and incubated in Dulbecco's modified Eagle's medium (Gibco BRL, Grand Island, NY, USA), containing 10% fetal bovine serum (Invitrogen, Camarillo, CA, USA). Each cell line was regularly authenticated by checking their morphology under the microscope.

RETRACTED

Male four-week-old specific pathogen-free BALB/C nude mice were purchased from Shanghai Research Center for Model Organisms and housed in laminar flow cabinets under specific pathogen-free conditions. The mice were feed with aseptic food and water. Animal studies conducted have been accordance with the guidelines of the NIH for the Care and Use of Laboratory Animals. The *in vivo* assay of nude mice was approved by the Institutional Animal Care and Use Committee of Shanghai General Hospital.

### Western blot

Cells were washed twice with PBS. Proteins were extracted from the cells using the BCA assay kit (Beyotime Biotechnology, Jiangsu, China) according to the manufacture's protocol, and were quantified with BSA as a standard. An equal sample volumes of protein (30 μg) were loaded for 10% SDS–PAGE, and transferred to a nitrocellulose membrane. After the blots were blocked by 5% non-fat milk, the target proteins were probed with primary antibodies at 4°C overnight. Then the membranes were washed three times and incubated with secondary antibodies. GAPDH was used as internal control protein. The following primary antibodies were used: anti-Smad4 (1:1000, Abcam, Cambridge, UK), anti-E-cadherin (1:50, Abcam, Cambridge, UK), anti-N-cadherin (1:1000, Abcam, Cambridge, UK) and anti-GAPDH (1:500, Abcam, Cambridge, UK).

### Total RNA extraction and qRT-PCR

The tissue specimens obtained from CRC patients after surgery were fixed in 10% formalin and embedded in paraffin. Total RNA were extracted from CRC cells using Trizol reagent (Invitrogen) and paraffin-embedded tissues using High Pure FFPE RNA Micro Kit (Roche) according to the manufacturer's instructions, respectively. After total RNA were reverse transcripted into complementary DNA which acted as the template for the amplification of RNA, real-time PCR was used for miR-20a-5p amplification and TaqMan Human miRNAs qPCR Quantitation Kit (Applied Biosystems, Foster City, CA, USA) for quantification following amplification. The small nuclear RNA U6 was used as normalized control. The Quantitative SYBR Green PCR Kit (Qiagen, Hilden, Germany) was used to quantify the Smad4 mRNA, E-cadherin and N-cadherin expression level respectively, GAPDH was used as the internal control. All the experiments were repeated at least triplicates [34, 37].

RETRACTED

### Luciferase reporter assay

To determine whether miR-224 directly targets the 3′-UTRs of Smad4, the wild-type or mutant Smad4 gene contained 3′UTR sequence with relative miR-20a-5p binding specific sequence was amplified and transfected into Dual Luciferase Reporter vector, and miR-20a-5p mimics, anti-miR-20a-5p or mutant-anti-miR-20a-5p mimics were cotransfected into relative CRC cells by Lipo2000 following the introductions. TK-Renilla plasmid was used as the control signal. The miR-20a-5p was mutated by changing Smad4 3′UTR binding site AAA to GGG (mut-miR-20a-5p) and mutant Smad4 3′UTR was formed with the mutant miR-520g binding site UUU to CCC. After 48 h, the cells were lysed and assayed using Dual-Luciferase^®^ Reporter Assay Kit (Promega) according to the manufacturer's instructions.

### Wound healing assay

Cells were cultured on 6-well plates forming single cell layer, and a straight wound line was made in the middle of the cell layer. After cultured for 48 h, cells that migrated into the wound line were observed. Images of cells along the wound line were taken by phase-contrast microscope (Nikon Digital ECLIPSE C1 system, Nikon Corporation, Japan).

### Migration and invasion assay

Transwell cell migration plates and Matrigel invasion chambers (8.0 μm pore size, BD Biosciences, Franklin Lakes, NJ, USA) were used to investigate the migration and invasion capability of different cells. Relative cells (5 × 10^5^ cells/ml) were seeded in serum-free medium into the upper chamber, and lower chamber added 20% FBS as chemo-attractant inducing cells invading towards the lower chamber. There was Matrigel coating layed on the upper chamber for invasion assay. After 8 h (migration assays) or 48 h (invasion assays), the cells that invaded through the membrane and adhered to the underside of the membrane were stained by 0.05% crystal violet and counted under microscope. All experiments were performed in triplicate, at least.

### Lentiviruses infection and cell transfection

Lentiviruses recombined with the indicated expression plasmids containing Smad4 overexpression, shSmad4 to attenuate the expression of Smad4 or negative control were obtained commercially (Genechem Co. Ltd., Shanghai, China). 5 × 10^5^ transducing units/mL of Smad4 overexpression lentiviruses particles were infected into HT29 cell and 5 × 10^5^ units/mL of Smad4 knockdown lentiviruses into HCT116 cells according to the manufacturer's protocols. Cultured cells were incubated with lentiviruses for 24 h, then replaced with fresh medium and incubated for another 48 h. Medium containing 1 μg/mL puromycin was used 7 days for selecting stable cell lines. HT29 and HCT-116 cells were transfected with constructed target gene (wt/mut-miR-20a-5p and wt/mut-Smad4) overexpression or knockdown plasmids using Lipofectamine 2000 (Invitrogen, Camarillo, CA, USA) according to the manufacturer's instructions, after cell transfection for 72 h, antibiotic selection (2 μg/ml puromycin) was selected for 5 days. For miR-20a-5p and Smad4 co-transfection, we constructed the plasmids with co-overexpression of miR-20a-5p and Smad4 or plasmids with co-silencing of miR-20a-5p and Smad4. The transfection method was consistent with that described above. The transfected efficiency of miR-20a-5p and Smad4 is showed in Supplementary Figure 1A and 1B.

RETRACTED

### Vector constructs

To generate the miR-20a-5p and Smad4 overexpression vector or knockdown vector and the corresponding negative controls, the open reading frame was amplified and cloned into the pcDNA3.0 vector. Luciferase constructs were generated by ligating oligonucleotides containing the wild type or mutant putative target site of the into the Psi-CHECK2 vector (Promega) downstream of the luciferase gene.

### Tumorigenesis in nude mice

Five homogeneous mice were divided into experimental and control group. The stable transfected cultured cells were harvested by trypsin digestion and washed with PBS, and resuspended with DMEM medium with 10% fetal bovine serum mixed. Next the cancer cells (1 × 10^6^/ml, 200 μl) were injected into tail vein of nude mice to evaluate the ability of liver metastasis. All mice were monitored every 7 days and were sacrificed 4 weeks later. The liver was exposed and grossly examined at necropsy, and then fixed in 10% formalin for HE staining. We counted the number of metastatic colonies macroscopically and calculated the average number of each group.

### TMA construction

TMA construction was undertaken as our previous report [32]. The expression of Smad4 was tested using standard immunohistochemical methods [33]. The Immunostaining was performed using primary antibodies anti-Smad4 (1:1000, Abcam, Cambridge, UK) incubated overnight at 4°C, and then incubated with HRP-conjugated anti-rabbit secondary antibodies (DakoCytomation, Glostrup, Denmark) for 30 min at room temperature.

Staining intensity of Smad4 was scored as follows: 0 for negative; 1, mild staining; 2, moderate staining; and 3, intense staining. The cell positive staining area was scored as follows: 0(0%), 1(1–25%), 2(26–50%), 3(51–75%) and 4(76–100%). The sum of intensity and extension was designated as the staining score, divided as follows: 0–2(negative expression); 3–4(weak positive expression); and 5–7 (strong positive expression). To avoid bias, two researchers blinded to patient information evaluated positive staining scores independently.

RETRACTED

### Statistical analysis

All data were presented as the mean±SD. The comparison between two groups was analyzed by students’ test. The correlation between miR-20a-5p and Smad4 expression levels was performed by calculating the Spearman correlation coefficient. Survival curves were analyzed using Kaplan– Meier method with log-rank test. Multivariate Cox-regression analyses were applied to evaluate the hazard ratio. All statistical analyses were performed using the SPSS 19.0 software (SPSS Inc, Chicago, IL). *P* < 0.05 was considered to be statistically significant.

## Supplementary Material


